# Two-Stream Retentive Long Short-Term Memory Network for Dense Action Anticipation

**DOI:** 10.1155/2022/4260247

**Published:** 2022-05-16

**Authors:** Fengda Zhao, Jiuhan Zhao, Xianshan Li, Yinghui Zhang, Dingding Guo, Wenbai Chen

**Affiliations:** ^1^School of Information Science and Engineering, Yanshan University, Qinhuangdao 066004, China; ^2^School of Information Science and Engineering, Xinjiang University of Science and Technology, Korla 841000, China; ^3^Key Laboratory for Software Engineering of Hebei Province, Yanshan University, Qinhuangdao 066004, China; ^4^Computing Division, School of Science and Technology, The University of Northampton, Northampton NN1 5PH, UK; ^5^Beijing Information Science and Technology University, School of Automaton, Beijing, China

## Abstract

Analyzing and understanding human actions in long-range videos has promising applications, such as video surveillance, automatic driving, and efficient human-computer interaction. Most researches focus on short-range videos that predict a single action in an ongoing video or forecast an action several seconds earlier before it occurs. In this work, a novel method is proposed to forecast a series of actions and their durations after observing a partial video. This method extracts features from both frame sequences and label sequences. A retentive memory module is introduced to richly extract features at salient time steps and pivotal channels. Extensive experiments are conducted on the Breakfast data set and 50 Salads data set. Compared to the state-of-the-art methods, the method achieves comparable performance in most cases.

## 1. Introduction

In recent years, great achievements have been made in the field of action recognition on RGB videos [1–3], depth, and RGB-D data [4–8]. However, these methods do not produce results until the action is complete. Action prediction aims to distinguish one or multiple actions when we only observe a partial video. It is a key to the success of many real-world applications, such as video surveillance, automatic driving, and efficient human-computer interaction.

Most current action prediction works forecast only one action several seconds earlier before it occurs [9–11] or distinguishes the action in an ongoing video [12–14]. However, in realistic applications, we often hope that the agents can forecast long-term actions. For example, a robot can interact with humans timely and efficiently, so the robot should understand the intention of humans and forecast the long-term actions of interactionists. However, long-term action anticipation raises great challenges as it is difficult to capture the relationships among long-term actions.

In this work, a novel model for dense action anticipation is introduced, which is called a two-stream retentive long short-term memory network (2S-RLSTM). To further understand what a video describes, this model exploits frame- and label-wise features at the same time. Our model, depicted in Figure 1, makes use of two types of inputs. One input focuses on frame-wise features extracted from RGB frames by pre-trained CNNs. The other input encodes label-wise features. On each stream, we use one LSTM layer to encode the input, which is followed by one more LSTM to preliminarily analyze sequence information. Then, the features are concatenated and fed into the retentive memory module. This module consists of a memory neural network and a channel-wise attention network. As inspired by the work of [15, 16], we utilize a memory neural network to extract features at salient time steps of the video. Recently, Wang et al. [17] prove that it is beneficial for capturing key information to avoid mapping features into low-dimensional spaces and increase interaction among features. Inspired by this work, we use a channel-wise attention network to capture information in key channels of the model. Finally, a fully connected layer is utilized to make classification and regression.

As evidenced by the experiments on the Breakfast data set [18] and 50 Salads data set [19], we prove that 2S-RLSTM helps improve the ability to forecast a series of actions and their duration and outperforms several state-of-the-art approaches for dense action anticipation by a relative increase in terms of accuracy.

The rest of this paper is organized as follows: Section 2 describes recent studies related to our work.  Section 3 introduces several crucial components of our model.  Section 4 reports and analyses the results of our method. The conclusion of this paper is given in Section 5.

The major contributions of this work are summarized as follows: (1) we propose a retentive memory module to capture relationships among long-term actions and (2) a new two-stream model to solve dense action anticipation and achieve comparable performance to the state-of-the-art methods.

## 2. Related Work

Although action recognition has achieved impressive results, it is limited to post-event analysis applications. On the contrary, action prediction methods can be used for pre-event analysis. These approaches for action prediction are divided into three main categories: early action prediction, sparse action anticipation, and dense action anticipation.

### 2.1. Action Recognition

Prior efforts, such as cuboids [20, 21], 3D HOG [22], SIFT [23], and dense trajectory [24], address the task of action recognition based on hand-crafted features. In recent years, methods based on deep learning have gained increased attention. Tran et al. [3] propose a C3D network to evolve time information in convolutional neural networks. Carreira et al. [1] also expand 2D convolution to 3D convolution and propose a large data set, the Kinetics data set. To some extent, a large data set solves the problem of being “data-hungry.” Hara et al. [2] design a deep 3D convolutional neural network, which is suitable to process the Kinetics data set.

Meanwhile, with the appearance of depth cameras, research on skeleton data have become gradually popular. Yan et al. [25] utilize graph convolutional networks to extract spatial features and temporal dynamics jointly. Considering the relationships of relatively remote joints, Li et al. [4] propose the A-link inference module to capture latent information among remote joints. Thakkar and Narayanan [8] divide the whole human skeleton into several parts and utilize graph convolution on each part. The work in [5] firstly describes the skeleton as a directed acyclic graph and allocates an adaptive graph topological structure to the skeleton. In their training process, the information on joints and bones is updated iteratively. Based on this work, Shi et al. [6] further take advantage of the second-order information, such as the length and direction of bones of skeleton data, which is naturally more informative and discriminative for action recognition. Si et al. [7] capture features in discriminative joints with an attention module and, in the meantime, employ temporal average pooling to reduce computation to some extent.

All these methods intend to extract valuable information in a complete data sequence, which is a kind of post-event classification, while action anticipation aims at distinguishing an action in an ongoing action sequence or forecasting one action, also perhaps several actions, before any of them occurs.

### 2.2. Action Prediction

In contrast to action recognition, early action prediction aims at predicting an action as early as possible in an ongoing video. This task is confronted with the challenge that a partial video contains insufficient information compared with a complete video.

Recently, various methods have been devoted to this task. Lan et al. [26] introduce a max-margin architecture to inference actions. Hu et al. [27] intend to learn a soft label for different progress levels of a video. Hence, full and partial videos can be learned in a unified regression framework. Aliakbarian et al. [12] jointly take advantage of context-a and action-aware information in each frame. Then the information is sent to multistage LSTM architecture to analyze the temporal dynamics of the video. Besides, a novel loss is used to ensure the accuracy of action classification at an early stage in a video. A novel knowledge distillation framework for early action prediction is introduced by the work in [14], which contains a student model, a teacher model, and a teacher-student learning block for distilling knowledge from teacher to student. Kong et al. [28] propose an adversarial action prediction network based on variational autoencoder and adversarial learning to jointly learns features and classifiers and generate the features particularly optimized for action prediction.

Unlike early action prediction, sparse anticipation aims at predicting one action in a video before it occurs. Sparse anticipation raises new challenges. It not only needs to analyze the observation but also needs the relationship among actions. Miech et al. [29] fuse a purely anticipatory model, which anticipates action directly from visual inputs, with a complementary model, which is constrained to reason about the present and then predicts one action a few seconds later. Ke et al. [11] concatenate encoded temporal information and action features to obtain global features of an action sequence, which ensures the accuracy of long-term prediction. On this basis, a skip connection with the last action and its encoded temporal information is added to the global features to jointly improve the accuracy of short- and long-term prediction.

Sparse anticipation presents another research route that is egocentric action anticipation. Egocentric action anticipation observes surroundings from a first-person perspective for some time and forecasts an action one second or several seconds later. Damen et al. [9] propose the first large-scale egocentric data set, the EPIC-KITCHENS data set. In the case of egocentric action anticipation, Damen et al. [9] utilize TSN [30] to predict an action one second before it occurs, which is regarded as a baseline for egocentric action anticipation on this data set. Furnari and Farinella [10] jointly extract appearance (RGB), motion (optical flow), and objects (object-based features) features to obtain rich information in observation. Subsequently, these features are fed into an attention module to fuse and adaptively attach different importance. Finally, these weighted features are summarized in an LSTM structure to predict actions at different moments.

### 2.3. Dense Action Anticipation

Different from sparse anticipation, dense anticipation aims at predicting an action sequence rather than a single action shortly. Sequence analysis becomes especially important in this task. Farha et al. [31, 32] use CNN and RNN to generate action sequences as well as their durations. Gammula et al. [15] embed memory neural networks into the LSTM network to obtain features at significant time steps. It is crucial to capture abundant features by an attention network in a long video if a good performance for action prediction is expected. Therefore, a retentive memory module is proposed to further capture features not only from salient time steps but also from pivotal channels and deal with the relationship among long-term actions.

## 3. Methodology

To model frame- and label-wise information, we introduce a two-stream architecture, which is shown in Figure 1. This model contains two types of inputs and finally extracts salient features by a retentive memory network. In this section, we first discuss our whole architecture and then analyze several crucial components of our model.

### 3.1. Two-Stream Retentive LSTM Network

Our goal is to forecast an action sequence and the duration of each action after observing a partial video. Specifically, the aim is to predict the action label of each frame after the observation. This procedure can be formulated as follows: let *X*_1_^*T*^={*x*_1_, *x*_2_,…, *x*_*T*_} be a video with *T* frames and *L*_1_^*T*^={*l*_1_, *l*_2_,…, *l*_*T*_} be action labels of the video. Given the observed frames *X*_1_^*t*^ and corresponding labels *L*_1_^*t*^, the target is to predict what will happen from frame *x*_*t*+1_ to the last frame *x*_*T*_pred__, where *x*_*T*_pred__ is the predicted frame count. Concretely, we want to infer the labels *L*_*t*+1_^*T*_pred_^={*l*_*t*+1_, *l*_*t*+2_,…, *l*_*T*_pred__} for each of the unobserved frames.

#### 3.1.1. Processing Strategy

Figure 2 illustrates the data processing strategy. Given an action sequence, we randomly cut each action except for the last action on the temporal axis. For each action in the observation, it can be represented as a two-tuple consisting of the action category and its observed length. At the predicting step, we observe the video before the cut line and predict a triple set, which consists of the label of the next action, the length of the next action before the cut line, and the remaining length of the current action. The observation visualization is shown in the “input representation” in Figure 2. It can be seen as a matrix. Each row of this matrix is a two-tuple mentioned above. The visualization of prediction results is shown in the “output representation” in Figure 2. It represents a matrix containing the elements of the triplet mentioned above. The results at the current step are added to the observation at the next step. The results are generated recursively until the length of the prediction reaches the expectation.

For label inputs, all the labels are encoded in a categorical form. More precisely, the encoded labels are in form of a composite vector, which consists of a one-hot vector and a length vector. The one-hot vector represents the class of action, while the length vector contains one element, which represents the remaining length of the current action. Due to high computational cost, for frame inputs, we only randomly choose several frames in observation as inputs. The targets are also encoded in a categorical form. Specifically, the targets consist of a one-hot vector and a compound length vector. The compound vector contains two elements. One represents the remaining length of the current action, and the other represents the length of the next action before the cut line.

#### 3.1.2. Action Anticipation Model

More formally, given the frame-wise inputs *X*_1_^*t*^={*x*_1_, *x*_2_,…, *x*_*t*_} and label-wise inputs *L*_1_^*t*^={*l*_1_, *l*_2_,…, *l*_*t*_}, we first transform the label inputs to categorical form *θ* in the way mentioned above as follows:

(1) $$\begin{array}{c} \theta =f_{\text{trans}}\left(L_{1}^{t}\right), \end{array}$$

where *f*_trans_(·) denotes the transform function that encodes label inputs to categorical form.

For frame-wise inputs *x*_*t*_, we use pre-trained CNNs to extract features from each frame. Here, we utilize ResNet50 [33] pre-trained on ImageNet [34] except for the last fully connected layer as our image feature extractor. Hence, we get a feature sequence *β* of observation.

As the categorical label information *θ* is a sparse matrix, it may be suitable for deep learning architecture. We take advantage of an LSTM layer to encode *θ*. Corresponding to this operation, an LSTM layer is also used to encode *β* in the frame-wise stream. The encoded sequences are defined as *θ* ′ and *β*′, respectively.

As is well known, an LSTM is beneficial to deal with sequence information. Thus, as shown in Figure 1, we exploit an LSTM to preliminarily analyze sequence features in each stream. Then we obtain preliminary features *α*, *γ* of the frame- and label-wise sequence, respectively, as follows:

(2) $$\begin{array}{c} \alpha =f_{LSTM}^{l}\left(\theta \prime \right),\\ \gamma =f_{LSTM}^{x}\left(\beta \prime \right), \end{array}$$

where *f*_*LSTM*_^*l*^(·) and *f*_*LSTM*_^*x*^(·) represent LSTM layers for analyzing preliminary sequence information in label stream and frame stream, respectively.

Then *α* and *γ* are concatenated to form a multimedia feature *ε*. This feature is fed into a retentive memory module to capture key information after such a long observation. This module consists of a memory neural network and a channel-wise attention network. Compared to LSTMs, a memory neural network is beneficial to capture the features in a long video. Thus, a memory neural network is utilized to capture the features in key time steps. Besides, to get further attended features, a channel-wise attention network is used to capture the features in pivotal channels. These procedures can be formulated as follows:

(3) $$\begin{array}{c} \omega =f_{\text{Atten}}\left(\text{concat}\left(\alpha ,\gamma \right)\right), \end{array}$$

where concat(·) denotes a function that concatenates the preliminary features, *α* and *γ*. Then, the concatenated feature is fed into the retentive memory module *f*_Atten_ and finally gets a salient feature *ω*. It is followed by a fully connected layer to discriminate the final output *y* in categorical form. The procedure can be formulated as follows:

(4) $$\begin{array}{c} y=f_{FC}\left(\omega \right), \end{array}$$

where *f*_*FC*_(·) represents the final fully connected layer. *y* is the output vector that consists of a one-hot vector and a compound vector. The one-hot vector represents the category of the next action. The compound vector includes two elements. One represents the remaining length of the current action. The other represents the length of the next action before the cut line.

For the loss function, because the output vector is a compound vector, a part of which requires classification and the other part wants regression, we deal with the output as follows:

(5) $$\begin{array}{c} L=-\text{log}\hat{a}+{\left(p_{n}-{\hat{p}}_{n}\right)}^{2}+{\left(p_{c}-{\hat{p}}_{c}\right)}^{2}, \end{array}$$

where $\hat{a}$ denotes the predicted vector for classification, which is used for the cross-entropy loss. *p*_*n*_ is the real length of the next action before the cut line, while ${\hat{p}}_{n}$ is the estimated one. Similarly, *p*_*c*_ is the real remaining length of the current action, while ${\hat{p}}_{c}$ is the estimated. Both ${\hat{p}}_{n}$ and ${\hat{p}}_{c}$ are applied to the mean squared error.

### 3.2. Retentive Memory Module

As the videos are usually too long to focus on key information, a retentive memory module is proposed to capture salient features. As shown in Figure 1, the module consists of a memory neural network and a channel-wise attention network. The preliminary features of both two streams are connected. Then the connected feature is fed into the retentive memory module. In this module, a memory neural network is utilized to deal with the features in key time steps of a video, and a channel-wise attention network is used to capture the features in pivotal channels.

Inspired by the work in [16], a memory neural network is adapted after the concatenation of preliminary features. The memory neural network consists of four main components: read operation *f*_*r*_, compose operation *f*_*c*_, write operation *f*_*w*_, and an encoding memory *M* ∈ *R*^*N*×*L*^, where *N* is the dimension of features and *L* is the length of memory. The architecture of the memory neural network is depicted in Figure 3.

The memory is initialized by the feature *ε* that is concatenated by the preliminary features, *α* and *β*. More formally, we initialize the memory *M* by *ε* directly, which can be formulated as follows:

(6) $$\begin{array}{c} M=\varepsilon . \end{array}$$

Then, these features are analyzed at each time step sequentially. For each time step, a read function is utilized to generate a query *q*_*t*_. Query *q*_*t*_ maps each slot by calculating the inner product and generates a series of association scores. Afterward, we normalize these scores with the softmax function without violating their orders and obtain a score vector *Z*. The score vector *Z* means the degree of importance of each slot. Thus, we take the weighted sum of all slots and get an attended vector *m*_*t*_. These procedures can be formulated as follows:

(7) $$\begin{array}{c} q_{t}=f_{r}\left(\varepsilon \right),\\ Z=\text{softmax}\left(q_{t}^{T}M\right),\\ m_{t}=Z^{T}M. \end{array}$$

Let *ε*_*t*_ denote the feature at time *t* in the original feature. In compose operation, we concatenate the feature *ε*_*t*_ and *m*_*t*_ and feed it into a multilayer perceptron:

(8) $$\begin{array}{c} c_{t}=f_{mlp}\left(\delta_{t},m_{t}\right), \end{array}$$

where *f*_*mlp*_(·) is a multilayer perceptron with a hidden layer.

In the write operation, we map *c*_*t*_ into output space. Finally, we update the memory space with a new representation:

(9) $$\begin{array}{c} h_{t}=f_{w}\left(c_{t}\right),\\ M^{t}=M^{t-1}⊙\left(1-z_{t}^{Τ}\right)+h_{t}⊙z_{t}^{Τ}, \end{array}$$

where ⊙ denotes element-wise product. Finally, we extract *c*_*t*_ at the last time step and feed it into the channel-wise attention network.

After obtaining salient features at each time step, we hope to further capture the features from pivotal channels. Inspired by the work in [17], we utilize a channel-wise attention network to enhance the critical information of pivotal channels in *c*_*t*_, which is generated by equation (11). Let us represent *c*_*t*_ as *c*. More formally, given an output feature *c* ∈ *R*^*K*^, the channel-wise attention network can be formulated as follows:

(10) $$\begin{array}{c} \eta =\sigma \left(Wc\right), \end{array}$$

where *W* denotes a parameter matrix in the shape of *K* × *K*. *σ* is a sigmoid function. In detail, *W* can be defined in form of *W*′ as shown in (11):

(11) $$\begin{array}{c} W{\;}^{\prime }=\left[\begin{array}{cccccccc} w_{1}^{1} & w_{1}^{2} & \cdots & 0 & 0 & \cdots & 0 & 0\\ 0 & w_{2}^{2} & \cdots & \vdots & w_{2}^{H+1} & \cdots & 0 & 0\\ \vdots & \vdots & \ddots & \vdots & \vdots & \ddots & w_{K-1}^{K-1} & 0\\ 0 & 0 & \cdots & 0 & 0 & \cdots & w_{K}^{K-1} & w_{K}^{K} \end{array}\right], \end{array}$$

where *w*_*i*_^*j*^ denotes the elements located at row *i* and column *j* in the parameter matrix. *W*′ involves *K* × *H* parameters. However, smaller *H* means features will be mapped into a lower-dimensional space, which may harm performance. Thus, an appropriate value for *H* can reduce the computational effort without seriously affecting the performance of the model. If different channels share weights, the parameter matrix *W*′ evolves *W*′, and *w*_*k*_ represents the shared parameter at row *k*.

(12) $$\begin{array}{c} W{\;}^{\prime \prime }=\left[\begin{array}{cccccccc} w_{1} & w_{1} & \cdots & w_{1} & 0 & \cdots & 0 & 0\\ 0 & w_{2} & \cdots & w_{2} & w_{2} & \cdots & 0 & 0\\ \vdots \; & \vdots \; & \ddots & \vdots \; & \vdots \; & \ddots & w_{K} & 0\\ 0 & 0 & \cdots & 0 & 0 & \cdots & w_{K} & w_{K} \end{array}\right]. \end{array}$$

Such a strategy can be readily implemented by a fast 1D convolution with a kernel size of *H*:

(13) $$\begin{array}{c} \eta =\sigma \left(C1\;D\left(c\right)\right), \end{array}$$

where *C*1  *D*(·) denotes a fast 1D convolutional network.

## 4. Experiment

In this section, we first compare our method with some state-of-the-art techniques on the task of dense action anticipation and then analyze several crucial components of our model. We also introduce implementation details and evaluation metrics in our experiments.

### 4.1. Data Set

The Breakfast data set [18] is a large-scale data set, which contains 1,712 video samples and consists of 48 action classes collected by 52 subjects. Each video sample contains a broad set of activities about preparing breakfast in daily life such as preparing milk, pancake, and tea, with an average length of 2.3 minutes and an average of 6 action instances. It is a challenging data set due to its large diversity of actions, long-range of videos, and variations of the camera's view angle. In our experiments, we follow the training/test split rules in [32]. Thus, the data set is divided into 4 parts. The first part is served as a test set, which contains 252 videos interpreted by 13 participants from P03 to P15. The other three parts are served as a training set, which contains 1,460 videos interpreted by 39 participants from P16 to P54.

The 50 Salads data set [19] contains 50 videos and consists of 17 action classes. It captures 27 people preparing salads, and each participant performs twice at random. Because of data loss, the videos of two participators, P08 and P12, are removed from the data set. Each video contains more than 7,000 frames, and many have more than 10,000 frames. In each video of this data set, the action sequence similarity is low, with similar actions only in the beginning part of the action and almost different actions in the back part. This increases the difficulty of supervised learning and brings great challenges to dense action anticipation. In our experiments, the 50 Salads data set is divided into 2 parts. The first part is served as a test set, which contains 10 videos interpreted by 5 participants from P13 to P17. The other part is served as a training set, which contains 40 videos interpreted by the other 20 participants.

### 4.2. Evaluation Metric

We follow the evaluation metric in [32], which is called mean over classes. This evaluation metric is formulated as follows:

(14) $$\begin{array}{c} MoC=\frac{1}{C}\sum_{i=1}^{C}\frac{l_{i}^{R}}{l_{i}^{R}+l_{i}^{W}}, \end{array}$$

where *C* is the number of action classes involved in the forecasting process. *l*_*i*_^*R*^ denotes the number of right labels of class *i*, while *l*_*i*_^*W*^ denotes the number of wrong labels of class *i*. The labels here refer to the label of each frame. The length of the action is expressed as the number of consecutive labels. This evaluation metric is a pretty restricted criterion due to its coefficient. Specifically, *MoC* represents the mean accuracy of classes involved in predicting process. In other words, if the accuracy of one class becomes low, *MoC* will decrease fiercely. Therefore, *MoC* can be high only if the accuracy of each action class is high.

### 4.3. Comparison to the State-of-the-Art

Our approach is compared to some state-of-the-art dense action anticipation approaches, and the results of experiments are reported as shown in Tables 1 and 2. There is no agreement on the proportion of frames that are observed or predicted, so we follow the experiment settings in [32] and forecast 10%, 20%, 30%, and 50% after observing 20% and 30%, respectively. The evaluation metrics of all experiments are those described in formula (14). The error criteria of the experiments are introduced in formula (5). As evidenced by the results in Tables 1 and 2, our method outperforms several state-of-the-art dense action anticipation approaches by a relative increase in accuracy in most cases.

For the label stream, we utilize the ground truth as input. As shown in Tables 1 and 2, our method improves the accuracy by approximately 5% in most items compared to CNN and RNN. During the training process, we noticed that our model converged much faster than RNN, which only utilizes the information of labels. It is because the frame stream provides abundant and detailed visual information to help the model understand what happens in the scenes. Besides, the label stream informs the model of what happens in the form of abstract language, so it may study better and faster from both two streams than from only label inputs. Furthermore, the key information of both two streams is captured by the retentive memory module to improve video comprehension ability.

However, on the 50 Salads data set, the accuracy of 2S-RLSTM when the observation ratio is 30% is not as high as when the observation ratio is 20%. The actions of the performers are arbitrary, and only the first few actions have a reference between the training set and the test set. When the observation ratio is 30%, we usually cannot find the action sequence similar to the predicted part in the training set, so it is difficult to predict the correct category of movements. Compared to CNN, our method has worse performance when observing 30% and predicting 50%. This is because our method operates iteratively, with errors generated in the current step accumulating into the next prediction. We find that the short-term prediction effect is inferior to RNN when the observation ratio is 30%. It is due to the difference in the action order between the training set and the test set after 30% observation and the lack of large empirical data. And then the information from the video frames facilitates the miscalculation. In these cases, the model is easy to make wrong judgments on the action category. But, if enough appropriate data is available to learn, the model can make an accurate prediction about future sequences of actions.

### 4.4. Analysis

In this section, we provide a detailed analysis of several components of our model on the Breakfast data set. For a fair comparison, we design a baseline composed of two LSTM layers and a fully connected layer, only involving the label stream.

To evaluate the frame stream, we add one more branch that consists of a ResNet50 [33] and two LSTM layers with the same dimension to the baseline. These features of both two streams are concatenated before the fully connected layer. The final output is generated by the fully connected layer. The evaluation results on the Breakfast data set are shown as 2S-LSTM in Table 3.

As evidenced by the results, the frame stream improves the performance of the model compared to the baseline. According to this case, we believe that RGB frames can provide abundant features for understanding the present and predicting the future reasonably. Specifically, an action may consist of several subactions. For example, “pour milk” may consist of “take up a milk carton,” “tilt the milk carton,” “pour milk from the milk carton,” and “put the milk carton on the table.” However, if we only use the information of labels, the information of subactions will not be used at all because the model may only know “pour milk” if we only feed information of labels to the model. Therefore, the frame stream provides detailed information to the model.

We then evaluate the retentive memory module that consists of a memory neural network and a channel-wise attention network, shown as L-CLSTM in Table 3. To this end, we first add the channel-wise attention network before the fully connected layer to the baseline. The results of L-CLSTM show that the channel-wise attention network improves the performance slightly, which is a little beneficial to enhance information in pivotal channels. Besides, to prove the effectiveness of the memory neural network, a memory network is inserted before the channel-wise attention network based on L-CLSTM. As shown in L-RLSTM in Table 3, the results illustrate the advantages of focusing on salient features extracted from highlighted time steps. Furthermore, we find the performance of 2S-LSTM and L-RLSTM is similar. We hold the opinion that the frame stream and the retentive memory module improve the performance from different aspects. Frame stream offers detailed information about subactions, while the retentive memory module captures salient information at prominent time steps and pivotal channels.

### 4.5. Limitations

In this section, the limitations of the proposed method will be discussed. Although the proposed method achieves comparable results, it has many obvious limitations. One of the limitations is that the approach relies on fine-grained action annotations. This requires explicit action labels for each frame of the observed video. However, in the real world, such fine-grained action annotations are difficult to obtain. Therefore, weakly supervised learning is a solution and a future research direction.

Another limitation is that the model has heavy components. In the task of action prediction, due to the limitation of the processing performance and storage space of some mobile devices, there are certain demands on the calculation speed and space size of the model. In the part of feature extraction, this model uses a ResNet50. And, in the part of feature analysis, the model is composed of a large module, which is termed the “retentive memory module.” The parameter amount of this model is about 40.44 M, and the calculation amount is about 26.59 G FLOPS. In addition, the computational burden of RGB image processing is relatively heavy. Therefore, a lightweight framework for fast data processing is necessary and is the future research direction.

## 5. Conclusion

In this paper, a novel method is proposed to predict a series of actions and their durations after observing a partial video. This model processes low-level features extracted from RGB videos and high-level features extracted from labels simultaneously. Moreover, to fully capture salient features in the long-range videos, a retentive memory module is utilized. This module extracts the features not only from salient time steps but also from pivotal channels. Finally, with extensive experiments on the Breakfast data set and 50 Salads data set, we verify the effectiveness of the model. The results show the method outperforms several state-of-the-art approaches for dense action anticipation by a relative increase in terms of accuracy in most cases. An efficient lightweight framework is the future research direction of this work.

## Figures and Tables

**Figure 1:** The architecture of 2S-RLSTM. Given a frame sequence and a label sequence, 2S-RLSTM can predict a series of actions and their durations in an iterative way.

**Figure 2:** Training samples are generated by cutting each action segmentation at a random split point. Each input sequence is a compound matrix of which each row consists of a double set, including the label and length of the observed action. Each target vector consists of a triple set, including the label of the next action, the remaining length of the current action, and the length of the next action before the cut line.

**Figure 3:** The architecture of a memory neural network. We extract features *c*_*t*_ in compose operation after the analysis of all time steps.

**Table 1:** Dense action anticipation performance comparison on the Breakfast data set.

Observation%	Prediction%	2S-RLSTM	CNN [32]	RNN [32]	Grammar [35]
20	10	65.04	57.59	60.35	48.92
	20	52.67	49.12	50.44	40.33
	30	50.42	44.03	45.28	36.24
	50	45.42	39.26	40.02	31.46

30	10	65.44	60.23	61.45	52.66
	20	54.59	50.14	50.25	42.15
	30	49.24	45.18	44.90	38.44
	50	46.03	40.51	41.75	33.09

**Table 2:** Dense action anticipation performance comparison on 50 Salads data set.

Observation%	Prediction%	2S-RLSTM	CNN [32]	RNN [32]	Grammar [35]
20	10	46.67	36.08	42.30	28.69
	20	33.32	27.62	31.19	21.65
	30	31.14	21.43	25.22	18.32
	50	19.76	15.48	16.82	10.37

30	10	39.96	37.36	44.19	26.71
	20	27.40	24.78	29.51	14.59
	30	21.23	20.78	19.96	11.69
	50	10.03	14.05	10.38	9.25

**Table 3:** Comparison of different architectures that are composed of different components.

Observation%	Prediction%	Baseline	2S-LSTM	L-CLSTM	L-RLSTM
20	10	54.26	59.45	57,24	58.35
	20	43.96	48.98	45.24	47.38
	30	41.86	46.19	42.81	46.01
	50	40.96	44.75	41.56	43.46

30	10	56.79	63.24	57.26	61.25
	20	51.87	52.69	52.67	53.61
	30	46.14	47.26	46.64	47.63
	50	42.69	44.85	43.79	44.51

## Data Availability

The experimental data and source files used to support the findings of this study have not been made available because of privacy.

## References

[1] Carreira J., Zisserman A. Quo vadis, action recognition? A new model and the Kinetics dataset.

[2] Hara K., Kataoka H., Satoh Y. Can spatiotemporal 3D CNNs retrace the history of 2D CNNs and ImageNet?.

[3] Tran D., Bourdev L., Fergus R., Torresani L., Paluri M. Learning spatiotemporal features with 3D convolutional networks.

[4] Li M., Chen S., Chen X., Zhang Y., Wang Y., Tian Q. Actional-structural graph convolutional networks for skeleton-based action recognition.

[5] Shi L., Zhang Y., Cheng J., Lu H. Skeleton-based action recognition with directed graph neural networks.

[6] Shi L., Zhang Y., Cheng J., Lu H. Two-stream adaptive graph convolutional networks for skeleton-based action recognition.

[7] Si C., Chen W., Wang W., Wang L., Tan T. An attention enhanced graph convolutional LSTM network for skeleton-based action recognition.

[8] Thakkar K., Narayanan P. J. (2018). *Part-Based Graph Convolutional Network for Action Recognition*.

[9] Damen D., Doughty H., Maria Farinella G. Scaling egocentric vision: the epic-kitchens dataset.

[10] Furnari A., Farinella G. What would you expect? Anticipating egocentric actions with rolling-unrolling LSTMs and modality attention.

[11] Ke Q., Fritz M., Schiele B. Time-conditioned action anticipation in one shot.

[12] Aliakbarian M. S., Saleh F. S., Salzmann M., Fernando B., Petersson L., Andersson L. Encouraging LSTMs to anticipate actions very early.

[13] Kong Y., Tao Z., Fu Y. Deep sequential context networks for action prediction.

[14] Wang X., Hu J.-F., Lai J.-H., Zhang J., Zheng W.-S. Progressive teacher-student learning for early action prediction.

[15] Gammulle P., Denman S., Sridharan S., Fookes C. (2019). Forecasting future action sequences with neural memory networks. *Proceedings of the 30th British Machine Vision Conference 2019, BMVC 201*.

[16] Munkhdalai T., Yu H. Neural semantic encoders.

[17] Wang Q., Wu B., Zhu P., Li P., Zuo W., Hu Q. ECA-net: efficient channel attention for deep convolutional neural networks.

[18] Kuehne H., Arslan A., Serre T. The language of actions: recovering the syntax and semantics of goal-directed human activities.

[19] Stein S., McKenna S. J. Combining embedded accelerometers with computer vision for recognizing food preparation activities.

[20] Dollar P., Rabaud V., Cottrell G., Belongie S. Behavior recognition via sparse spatio-temporal features.

[21] Fathi A., Mori G. Action recognition by learning mid-level motion features.

[22] Klaser A., Marszałek M., Schmid C. (2008). A spatio-temporal descriptor based on 3D-gradients. *British Machine Vision Association*.

[23] Scovanner P., Ali S., Shah M. A 3-dimensional sift descriptor and its application to action recognition.

[24] Wang H., Schmid C. Action recognition with improved trajectories.

[25] Yan S., Xiong Y., Lin D. (2018). *Spatial Temporal Graph Convolutional Networks for Skeleton-Based Action Recognition*.

[26] Lan T., Chen T.-C., Savarese S. A hierarchical representation for future action prediction.

[27] Hu J. F., Zheng W. S., Ma L., Wang G., Lai J., Zhang J. (2019). Early action prediction by soft regression. *IEEE Transactions on Pattern Analysis and Machine Intelligence*.

[28] Kong Y., Tao Z., Fu Y. (1 March 2020). Adversarial action prediction networks. *IEEE Transactions on Pattern Analysis and Machine Intelligence*.

[29] Miech A., Laptev I., Sivic J., Wang H., Torresani L., Tran D. Leveraging the present to anticipate the future in videos.

[30] Wang L., Xiong Y., Wang Z. Temporal segment networks: towards good practices for deep action recognition.

[31] Abu Farha Y., Gall J. Uncertainty-aware anticipation of activities.

[32] Farha Y. A., Richard A., Gall J. When will you do what? - anticipating temporal occurrences of activities.

[33] He K., Zhang X., Ren S., Sun J. Deep residual learning for image recognition.

[34] Russakovsky O., Deng J., Su H. (2015). ImageNet large scale visual recognition challenge. *International Journal of Computer Vision*.

[35] Richard A., Kuehne H., Gall J. Weakly supervised action learning with RNN based fine-to-coarse modeling.

